# GCN5 inhibition prevents IL-6-induced prostate cancer metastases through PI3K/PTEN/Akt signaling by inactivating Egr-1

**DOI:** 10.1042/BSR20180816

**Published:** 2018-11-30

**Authors:** Guangfeng Shao, Yuqiang Liu, Tianjia Ma, Lei Zhang, Mingzhen Yuan, Shengtian Zhao

**Affiliations:** 1 Department of Urology, The second hospital of Shandong University, Ji’nan, Shandong 250033, China; 2 Shandong Provincial Hospital, Ji’nan,Shangdong 250021, China; 3 Key Laboratory for Kindey Regeneration of Shandong Province, Ji’nan, Shangdong 250033, China; 4 Shandong University-Karolinska Institute Collaborative Laboratory for Stem Cell Research, Ji’nan,Shandong 250033, China

**Keywords:** Egr-1, GCN5, metastasis, proliferation, prostate cancer

## Abstract

General control non-derepressible 5 (GCN5) is ectopically expressed in different types of human cancer and association with the carcinogenesis, development, and poor prognosis of cancers. The present study was aimed to investigate the potential role and related mechanisms of GCN5 in IL-6–treated prostate cancer (PCa) cell. The results showed that an elevated GCN5 expression was stimulated by IL-6. Knockdown of GCN5 significantly inhibited IL-6–driven proliferation, migration, invasion, and epithelial-mesenchymal transition (EMT). Moreover, early growth response-1 (Egr-1) expression was elevated by IL-6 treatment and GCN5 siRNA down-regulated the expression of Egr-1. Furthermore, overexpression of Egr-1 attenuated the effects of GCN5 silence on cell proliferation, migration, invasion, and EMT in PCa. Besides, knockdown of GCN5 resulted in the down-regulation of p-Akt and up-regulation of PTEN, which was partly impeded by Egr-1 overexpression. The effects of GCN5 overexpression on cell proliferation and invasion were suppressed by LY294002, In conclusion, these data demonstrated the negative effect of up-regulated GCN5 in IL-6-induced metastasis and EMT in PCa cells through PI3K/PTEN/Akt signaling pathway down-regulating Egr-1 expression.

## Introduction

Prostate cancer (PCa) is the most frequently diagnosed cancer and the second leading cause of cancer-related death worldwide in male [1]. The high morbidity and mortality of PCa are mainly due to the distant metastases, in which the cancer cells spread from a primary organ to distal sites. Substantial evidence has demonstrated that inflammation also plays a critical role in the pathogenesis of PCa by regulating tumor microenvironment through releasing proinflammatory cytokines and growth factors, and thus modulating the tumor growth, progression, and metastasis [2–4]. Therefore, it is very important to understand the molecular pathway associated with metastasis and inflammation for improving approaches to therapy and prevention of PCa.

Interleukin (IL)-6 is a potent proinflammatory cytokine that exhibits functional pleiotropy in the regulation of growth, metastasis, and differentiation in numerous human cancers such as lung cancer, head and neck squamous cell carcinoma, breast, and PCa [5–8]. High level of IL-6 has been found in clinical specimens from PCa patients and PCa cell lines (PC3, DU145, and LNCaP et al), as well as in sera of patients with advanced PCa that is resistant to therapy [9]. Furthermore, the elevated IL-6 level has been reported to promote PCa growth and metastatic potential acquisition through modulating the cell proliferation, invasion, migration, and epithelial-mesenchymal transition (EMT) of PCa, while anti-IL-6-antibody showed a contrary effect [7]. In PCa, activation of STAT3 and IGF-1R signaling pathway by IL-6 has been indicated to be key molecular events in the progression and metastasis [10,11]. Thus, IL-6 is an important regulator in the tumorigenesis and development of PCa. However, the molecular mechanism of IL-6-induced EMT and metastasis in PCa has not been investigated thoroughly.

General control non-derepressible 5 (GCN5), also named KAT2A, is the first identified histone lysine acetyltransferase belongs to HAT superfamily. The involvement of GCN5 has been reported in a broad range of cellular processes including gene transcription, differentiation, DNA repair, nucleosome assembly, and cell cycle regulation [12–16]. In addition, it has also been manifested that GCN5 plays a role in cancer cell growth and development through increasing the stability of c-Myc and the translocated E2A-PBX1 oncoprotein [16–19]. However, the functional role and mechanism of GCN5 in the EMT and metastasis of PCa are still unclear. The aim of our current study is to evaluate the role of GCN5 in IL-6–stimulated PCa, we first determined the expression level of GCN5 after IL-6 treatment, and then the effects of silencing GCN5 on cell invasion, migration and EMT were evaluated. Finally, we further explored the potential mechanism that involved.

## Materials and methods

### Cell culture and treatment

The human PCa cell lines TSU, PC-3, LNCaP, and DU145 were purchased from the Cell Bank of Type Culture Collection of Chinese Academy of Sciences (Shanghai, China) and cultured in RPMI-1640 medium (Gibco-BRL, Rockville, MD, U.S.A.) plus 100 U/ml of penicillin, 100 mg/ml of streptomycin, and 10% FBS (Gibco-BRL) in a humidified atmosphere at 37˚C in 5% CO_2_. For IL-6 treatment, recombinant human (rh) IL-6 (R&D Systems, Minneapolis, MN, U.S.A.) was diluted in cell culture medium to a concentration of 20 ng/ml and used to maintain cells for 24 h.

### RT-qPCR

Cells were harvested, and total RNA was extracted using TRI-reagent (Sigma–Aldrich, St Louis, MO, U.S.A.) according to manufacturer’s protocol. About 2 μg of RNA was reversed to synthesize DNA using the Superscript II First Strand cDNA Synthesis Kit (Invitrogen, Carlsbad, CA, U.S.A.). Real-Time PCR was performed according to the manufacturer’s protocol of Fast Start Universal SYBR Green Master (Roche Diagnostics, Indianapolis, IN) using Applied Biosystem’s 7900 HT Real-Time PCR system.

### Western blotting

Total protein was prepared using ice-cold lysing buffer (50 mM Tris–HCl [pH 7.4], 1% NP-40, 0.1% SDS, 0.25% sodium deoxycholate, 150 mM NaCl, 1 mM EDTA, 1 mM PMSF, 1 lg/ml leupeptin, 1 μg/ml aprotinin, 1 μg/ml pepstatin, 1 mM Na3VO4, and 1 mM NaF). Protein concentration was determined using the Pierce BCA Assay Kit (Thermo Scientific). Equal amounts of protein were resolved by SDS/PAGE on 4–20% gels (Novex/Invitrogen, San Diego, CA) and transferred to a PVDF membranes. Then the membrane was blocked with 5% non-fat dry milk, followed by incubating with rabbit anti-BRD4(1:1000), rabbit anti-α-catenin (1:1000), rabbit anti-E-cadherin(1:1000), rabbit anti-Vimentin (1:1000), rabbit anti-N-cadherin (1:1000), rabbit anti-β-Catenin(1:1000), rabbit anti-CyclinD1(1:1000) and rabbit anti-c-myc(1:1000) antibodies, and HRP-conjugated mouse anti-rabbit secondary antibody(1:5000; Cell Signaling Technology, Danvers, MA, U.S.A.). The blots were visualized by enhanced chemiluminescence (Bio-Rad Laboratories, Hercules, CA). The intensity of the target proteins was normalized to the intensity of β-actin.

### Plasmids and siRNA transfection

The on-target plus siRNA for GCN5 (siGCN-1 and siGCN-2), and non-targetting control siRNA (NC), as well as pcDNA3.1 expression plasmids encoding Egr-1 (pcEgr-1) were purchased from Santa Cruz co (Santa Cruz, CA, U.S.A.). The pcDNA-Flag-GCN5 plasmids express human GCN5 or its corresponding mutant cDNA respectively with FLAG-tag using the cytomegalovirus immediate early promoter. LNCaP cells were planted into a six-well plate, siGCN5-1, siGCN5-2, pcEgr-1, and NC were transfected until the cells were 80% confluent according to the manufacturer’s instructions of Lipofectamins^TM^ 2000 (Invitrogen). The cells were further cultured for 24  h before supernatant was collected and cells lysed for transfection efficiency or other experimental analysis.

### MTT assay

In brief, cells (4 × 10^5^) were seeded in 96-well plates and 12, 24, 48, 72, or 96 h after, 5 mg/ml MTT was added and it was incubated for another 4 h. Then, cells were stained with 200 μl of DMSO. After that, the plate was read at 570 nm using a spectrophotometer (Beckman Coulter).

### Invasion assay

The cell invasive ability was performed using a BD BioCoat Matrigel Invasion Chamber (BD Biosciences, Piscataway, NJ, U.S.A.) according to the manufacturer’s protocol. In brief, the cultured cells (5 × 10^4^) treated with IL-6, siGCN5, and pcEgr-1 were seeded in serum-free RPMI-1640 medium in the matrigel-coated chamber inserts, and the lower chamber was filled with RPMI-1640 medium with 10% serum. After 24 h of incubation at 37°C, the non-invasive cells on the upper chambers were carefully removed with a cotton-tipped swab. The invading cells on the bottom chamber were fixed with 100% methanol and stained with 0.05% crystal violet, and counted under an immnofluorescence microscopy. Results were collected in five random microscopic fields per membrane in triplicate inserts.

### Migration assay

The migratory capacity of migration cells treated with IL-6, siGCN5, and pcEgr-1 was measured using Corning transwell inserts (BD Biosciences) with 8.0 μm pore polycarbonate membrane. 5 × 10^4^ cells were incubated in medium with 1% FBS in the top transwell chamber of the system and allowed to migrate for 48 h. After removing non-migrated cells from the upper chamber using a cotton swab, the cells were then fixed and stained with 0.05% crystal violet. The number of migrated cells was determined by counting in four fields/well with three wells/condition.

### Statistical analyses

Data were presented as the mean ± S.D. from at least three independent experiments. Statistical analyses were performed using the Student’s *t* test and one-way ANOVA. *P*<0.05 was considered statistically significant.

## Results

### IL-6–stimulated GCN5 expression in various PCa cell lines

The GCN5 mRNA and protein expression levels in human prostate carcinoma cell lines after IL-6 treatment were investigated using RT-qPCR and Western blotting assay. Results revealed that GCN5 mRNA expression level was significantly up-regulated by IL-6 stimulation in the whole PCa cell lines, in which LNCaP cell line showed a maximum induction (Figure 1A). The GCN5 protein expression level was also elevated in various PCa cells, with the biggest promotion in LNCaP cell line (Figure 1B).

**Figure 1:** GCN5 is up-regulated in IL-6–stimulated PCa cells Cells were cultured and then treated with IL-6 (20 ng/ml) for 24 h, (**A**) GCN5 mRNA expression was determined using RT-qPCR analysis. (**B**) The protein expression level of GCN5 was measured using Western blotting assay. The error bars represent the means ± S.D. of three independent experiments. *P<0.05 compared with control group.

### Knockdown of GCN5 inhibited proliferation in IL-6-induced PCa

Next, we investigated the effect of GCN5 on cell proliferation of LNCaP cell. GCN5 was efficiently silenced by siGCN5-1 and siGCN5-2 (Figure 2A). MTT assay was performed to determine the cell proliferation. As Figure 2B showed, IL-6 stimulation significantly promoted the cell proliferation, and down-regulation of GCN5 remarkably inhibited proliferation of LNCaP cells (Figure 2B).

**Figure 2:** Knockdown of GCN5 inhibited proliferation by IL-6–stimulated in PCa cells Cells were cultured and then treated with IL-6 (20 ng/ml) for 24 h, GCN5 siRNAs were then transfected and cultured for another 24 h. (**A**) The protein expression level of GCN5 was measured using Western blotting assay. (**B**) Cell proliferation was determined using MTT assay. The error bars represent the means ± S.D. of three independent experiments. *P<0.05 compared with control or NC. #*P*<0.05 compared with NC.

### Knockdown of GCN5 inhibited IL-6–driven migration, invasion, and EMT

As shown in Figure 3A & B, siGCN5-1 and siGCN5-2 mediated silence of GCN5 prevented IL-6-induced invasion and migration of PCa cells. Furthermore, knockdown of GCN5 repressed mesenchymal markers Vimentin, N-cadherin, and upr-egulated epithelial markers α-catenin and E-cadherin protein expression levels after IL-6 exposure (Figure 3C).

**Figure 3:** Knockdown of GCN5 inhibited metastasis and EMT induced by IL-6–stimulated in PCa cells Cells were cultured and then treated with IL-6 (20 ng/ml) for 24 h, GCN5 siRNAs were then transfected and cultured for another 24 h. (**A**) The number of invasive cells was counted and analyzed statistically by Matrigel Invasion Chamber assay. (**B**) The number of migrated cells was counted and analyzed statistically by transwell assay. (**C**) The protein expression levels of epithelial markers and mesenchymal markers were analyzed using Western blotting assay and representative blots are shown. The error bars represent the means ± S.D. of three independent experiments. *P<0.05 compared with the control or NC. #*P*<0.05 compared with the control or NC.

### Overexpression of Egr-1 attenuated the effects of GCN5 silence on PCa

Early growth response-1 (Egr-1) protein expression level was significantly impeded by GCN5 knockdown (Figure 4A). To explore the role of Egr-1 in IL-6–treated PCa cells, the Egr-1 overexpression plasmid was used, and the metastasis and EMT of PCa cells were analyzed. Results showed that overexpression of Egr-1 impeded the inhibited cell proliferation induced by siGCN5 (Figure 4B). Ectopic expression of Egr-1 attenuated the inhibitory effect of siGCN5 on invasion (Figure 4C) and migration (Figure 4D) of PCa cells. What’s more, the Western blotting assay manifested that overexpression of Egr-1 partly abrogated suppressive effect of siGCN5 on Vimentin protein expression (Figure 4E) and the promotional effect of siGCN5 on the E-cadherin protein expression (Figure 4F).

**Figure 4:** Overexpression of Egr-1 attenuated the effects of GCN5 silence in PCa Cells were cultured and then treated with IL-6 (20 ng/ml), GCN5 siRNA (siGCN5), and pcDNA 3.1 Egr-1 (pcEgr-1). (**A**) The protein expression level of Egr-1 was measured using Western blotting assay. (**B**) The cell proliferation was tested using MTT assay. (**C**) The number of invasive cells was counted and analyzed statistically by Matrigel Invasion Chamber assay. (**D**)The number of migrated cells was counted and analyzed statistically by transwell assay. The protein expression levels of epithelial markers (**E**) Vimentin and (**F**) E-cadherin were analyzed using Western blotting assay and representative blots are shown. The error bars represent the means ± S.D. of three independent experiments. *P<0.05 compared with Blank. #*P*<0.05 compared with NC. $*P*<0.05 compared with siGCN5.

### PI3K/PTEN/AKT signaling was involved in cancer growth and metastasis following GCN5 overexpression

Finally, we investigated the effects of GCN5 on PI3K/Akt signaling. Western blotting showed siGCN5 significantly decreased the protein expression level of Akt phosphorylation (p-Akt) and increased PTEN protein expression level, which were reversed by Egr-1 overexpression (Figure 5A). Meanwhile, pcEgr-1 remarkably increased the protein expression level of p-Akt and down-regulated the PTEN protein expression level (Figure 5A). These results indicate that siGCN5 inhibits Akt phosphorylation and activates PTEN. Furthermore, MTT assay results showed that pretreatment with the PI3K/Akt inhibitor, LY294002, rivalry suppressed pcGCN5 of IL-6-induced PCa cell proliferation and invasion (Figure 5B,C).

**Figure 5:** PI3K/PTEN/Akt signaling was a downstream effector of GCN5 in regulating PCa cell proliferation and invasion Cells were cultured and then treated with IL-6 (20 ng/ml), GCN5 siRNAs (siGCN5), pcDNA 3.1 Egr-1 (pcEgr-1), pcDNA-FLAG-GCN5 (pcGCN5). (**A**) The protein expression level of p-Akt, Akt, and PTEN were measured using Western blotting assay. (**B**) The cell proliferation was tested using MTT assay. (**C**) The number of invasive cells was counted and analyzed statistically by Matrigel Invasion Chamber assay. The error bars represent the means ± S.D. of three independent experiments. #*P*<0.05 compared with NC. $P<0.05 compared with siGCN5.

## Discussion

Although patients treated with chemotherapies display characteristic progression, the therapeutics of PCa were still impeded due to the complex molecular mechanism involved in the carcinogenesis, development, and metastasis of cancer. Blockade of the IL-6 signaling pathway has been regarded as a target for the therapy in variety of cancers. Monoclonal antibodies against IL-6 (Siltuximab) and the IL-6 receptor (IL-6R, Tocilizumab) have emerged as potential immunotherapies [20]. Recent advances in the investigation of cytokines in PCa suggested that IL-6 played an important role in the progression and metastasis of PCa and benign prostatic hyperplasia [21]. Thus, a deeper understanding of the involved molecular mechanisms underlying PCa development could help to build more efficient therapeutic strategies in the battle against PCa. The present study demonstrated that GCN5 is up-regulated in the IL-6–treated TSU, PC-3, LNCaP, and DU145 cells, which suggested a potential role of GCN5 in IL-6–treated PCa cell lines.

High expression of GCN5 was found in multiple types of human cancers. Chen et al [16] found that GCN5 was highly expressed in lung cancer, and its expression was positively linked to tumor size. Besides, overexpression of GCN5 significantly promoted cell growth of lung cancer. Majaz et al [22] reported that GCN5 was frequently overexpressed in human hepatocellular carcinoma tissues and cell lines, and silence of GCN5 inhibited cell proliferation, cell cycle progression, and xenograft tumor formation. The elevated GCN5 expression was also observed in colon cancer andurothelial carcinoma, in which GCN5 suppression reduced cell proliferation [18,23]. In the present study, knockdown of GCN5 prevented IL-6-induced invasion and migration of PCa cells, which was in accordance with the result of Li et al [17] who reported GCN5 has a positive effect on cell migration in breast cancer. Besides, the study of Wang et al [24] suggested an involvement of GCN5 in MDC1-regulated cell growth and migration. Activation of an EMT program has been proposed as the critical mechanism for the acquisition of invasiveness and metastasis. The present study observed that GCN5 inhibition reversed the accelerative effect of IL-6 on EMT in PCa. It has been well investigated that IL-6–stimulated metastasis through induction of EMT. Therefore, GCN5 plays an important role in promoting EMT and metastasis of IL-6 in PCa.

GCN5, as a histone acetyltransferase, has been famous for its function in transcription regulation. Recently, it has been reported that GCN5 inhibition is able to activate transcription factor Egr-1 in neurone [25]. Egr-1 is an important regulator of cell proliferation, apoptosis, metastasis, and EMT in the progression of kinds of cancers including PCa and functions as a tumor suppressor in various of cancers [26–29]. Egr-1 is induced by many different stimuli such as growth factors, environmental stresses and cytokines [30–32]. Inhibition of Egr-1 has reported to inhibit apoptosis and enhance cell proliferation of PCa [33,34]. Ma et al [35] indicated that targetted knockdown of Egr-1 inhibited IL-8-induced tumor colony formation and invasion of PCa. Interestingly, in the present study, we found Egr-1 was up-regulated by IL-6 stimulation, and inhibition of Egr-1 partly reversed the modulation of GCN5 in cell proliferation and metastasis of IL-6-induced PCa cells. Therefore, we speculate that GCN5 might promote IL-6-induced cell proliferation, invasion, migration, and EMT through down-regulating Egr-1 in PCa.

The PI3K/PTEN/Akt signaling is a key regulator of cell proliferation, apoptosis, survival, differentiation, motility, and metabolism [36]. Accumulating evidences in the literature have shown that the PI3K/PTEN/Akt signaling pathway is critical regulator in cell apoptosis, proliferation, invasion, metastasis and prognosis of cancers [37,38]. As a tumor suppressor, PTEN is known as a direct antagonist of PI3K and negatively regulates the Akt signal pathway. Our findings indicated that knockdown of GCN5 resulted in the down-regulation of p-Akt and up-regulation of PTEN, which was partly impeded by Egr-1 overexpression. Furthermore, the effect of GCN5 overexpression on cell proliferation and invasion rivalry suppressed by LY294002, confirming that GCN5 acts its role in PCa partly through the PI3K/PTEN/Akt signaling pathway.

In conclusion, our results manifested the negative effect of up-regulated GCN5 in IL-6-induced metastasis and EMT in PCa cells by down-regulating Egr-1through PI3K/PTEN/Akt signaling pathway. These findings elucidate the anticancer effects of GCN5 in PCa and targetting GCN5 may have the potential to block metastasis.

## Abbreviations

EMT: epithelial-mesenchymal transition
GCN5: general control non-derepressible 5
IL: interleukin
PCa: prostate cancer
PTEN: phosphatase and tensin homolog deleted on chromosome ten
PVDF: polyvinylidene fluoride
RT-qPCR: quantitative reverse transcription PCR
